# Unraveling the causative connection between urticaria, inflammatory cytokines, and mental disorders: Perspectives from genetic evidence

**DOI:** 10.1111/srt.13906

**Published:** 2024-09-19

**Authors:** ZhiRong Liu, YuanYing Wang, ShiHao Wang, JiaXin Wu, Cui Jia, Xuan Tan, XinLian Liu, XinWei Huang, LuShun Zhang

**Affiliations:** ^1^ Department of General Surgery Chengdu Second People's Hospital Chengdu China; ^2^ Graduate School Chengdu Medical College Chengdu China; ^3^ School of Biological Science and Technology Chengdu Medical College Chengdu China; ^4^ Development and Regeneration Key Laboratory of Sichuan Province Institute of Neuroscience Department of Pathology and Pathophysiology Chengdu Medical College Chengdu China; ^5^ Shanghai Key Laboratory of Anesthesiology and Brain Functional Modulation Clinical Research Center for Anesthesiology and Perioperative Medicine Translational Research Institute of Brain and Brain‐Like Intelligence Shanghai Fourth People's Hospital School of Medicine Tongji University Shanghai China

**Keywords:** causal association, inflammatory cytokines, Mendelian randomization, mental disorders, urticaria

## Abstract

**Background:**

The genetic association between urticaria and mental disorders and whether inflammatory cytokines mediate this process remains unclear.

**Materials and methods:**

A Mendelian randomization (MR) approaches to elucidate the causal relationship between urticaria and mental disorders and to validate the mediation of inflammatory cytokines. Genome‐wide association study (GWAS) databases used were obtained from Psychiatric Genomics Cooperation (PGC), GWAS Catalog, and FinnGen Consortium. Our study was conducted using inverse variance weighted (IVW) and Bayesian weighted MR (BWMR) methods for joint analysis.

**Results:**

The MR results showed that urticaria increased the risk of attention deficit hyperactivity disorder (ADHD) (odds ratio [OR] = 1.088, 95% confidence interval [CI]: 1.026–1.154, *p* = 0.0051); cholinergic urticaria increased the risk of bipolar disorder (BD) (OR = 1.012, 95% CI: 1.001–1.022, *p* = 0.0274); dermatographic urticaria increased the risk of ADHD (OR = 1.057, 95% CI: 1.005–1.112, *p* = 0.0323); idiopathic urticaria increased the risk of schizophrenia (SCZ) (OR = 1.057, 95% CI: 1.005–1.112, *p* = 0.0323); other unspecified urticaria increased the risk of ADHD (OR = 1.085, 95% CI: 1.023–1.151, *p* = 0.0063). We found that eight inflammatory cytokines were negatively associated with mental disorders and seven inflammatory cytokines were positively associated with mental disorders. Finally, our results suggested that inflammatory cytokines do not act as mediators between urticaria and mental disorders.

**Conclusions:**

Our study reveals a causal relationship between urticaria and the increased risk of mental disorders. We suggest that the treatment of urticaria could incorporate psychiatric interventions and mental health assessment of patients.

## 1 INTRODUCTION

Urticaria, a syndrome characterized by wheals (hives), angioedema, or both, is a very common inflammatory skin disease in daily life.^1^ It is caused by mast cell activation and degranulation, which subsequently promotes the release of histamine and other mediators, and it can be spontaneous or induced by various factors.^1^ According to the duration of the disease, urticaria can be classified into two clinical types: acute and chronic. Acute urticaria is lasts less than 6 weeks, and usually associated with infection, food, or drug ingestion. Chronic urticaria (CU) can be categorized as chronic spontaneous urticaria (CSU, where no specific trigger can be found) or chronic induced urticaria (CIndU, induced by a definite stimulus) based on the presence or absence of a definite trigger, and the duration of the disease is usually more than 6 weeks.^2^, ^3^ CIndU can also be categorized into physical urticaria, which may be caused by friction, touch, vibration, cold or heat, pressure, or sunlight exposure, and non‐physical urticaria, which includes contact urticaria and cholinergic urticaria.^4^ Urticaria may universally manifest itself in all areas of the skin, the resultant scratchy rash exhibits a tendency to worsen at night and lasts long before subsiding. Due to the unbearable torment of itching, some urticaria patients may be accompanied by systemic symptoms such as fever, fatigue, gastrointestinal disturbances, and arthralgia.^5^, ^6^ And these symptoms can lead to a dramatic reduction in the quality of life of the patient and cause stress, sleep disturbances, negative emotions, low mood, sadness, anxiety, and depression.^7^, ^8^, ^9^, ^10^ The pathophysiology of urticaria is especially complicated because there is evidence of a reciprocal relationship between the immune system and the central nervous system (CNS),^11^, ^12^ in which inflammatory cytokines may cross the blood–brain barrier (BBB) and trigger neuro‐immune processes linked to mood and behavior regulation during the atopic reaction.^18^, ^19^

However, some studies have found results that do not support a link between urticaria and mental disorders, so the association between urticaria and mental disorders remains a topic of controversy.^13^, ^14^, ^15^ Actually, those different results may lie in following reason, the data used in those studies may be affected by heterogeneity and confounding factors (e.g., age, gender, and comorbidity) that reduce the reliability of the data. In addition, genetic, biological, or environmental risk factors may be common or overlapping and lead to confounding effects. Therefore, a more rigorous methods is needed to validate the relationship between the urticaria and mental disorders.

Mendelian randomization (MR), a new method of genetic epidemiological analysis, is widely adopted in researches. The method is designed to follow Mendel's second law of inheritance, which states that “alleles from parents are randomly assigned to offspring.”^16^ If the phenotype is determined by the genotype, then the phenotype will link the genotype to the disease.^17^, ^18^Therefore, in order to deduce the relationship between phenotype and disease, genotype might be employed as instrumental variables (IVs).^19^, ^20^ In addition, genotypes cannot be altered by disease, MR analyses are less susceptible to confounding, reverse causation, and measurement error than traditional observational studies.^17^, ^21^ This study will explore the genetic associations between urticaria and mental disorders using a two‐sample MR approach with urticaria (idiopathic urticaria, allergic urticaria, dermatographic urticaria, contact urticaria, urticaria due to cold and heat, cholinergic urticaria, other and unspecified urticaria) as exposure and four mental disorders (attention deficit hyperactivity disorder [ADHD], bipolar disorder (BD), major depressive disorder (MDD), and schizophrenia [SCZ]) as outcome. Subsequently, we explored whether inflammatory cytokines could act as mediators to influence the genetic causal association between urticaria and mental disorders.

## 2 METHODS

### 2.1 Study design

The MR approach is based on integrating datasets from large genome‐wide association studies (GWAS), using single nucleotide polymorphisms (SNPs) as IVs to infer causal relationships between exposures and outcomes^22^, ^23^. Since this study involved the analysis of publicly available summary data, no informed permission nor ethical approval were needed for it. Figure 1 briefly summarizes the design process of this MR study, which consisted of a total of three parts:

1. Analysis of causal effects exploring (and its seven subtypes) and four mental disorders (Figure 1: Step 1).
  ① Exposures: urticaria, idiopathic urticaria, allergic urticaria, dermatographic urticaria, contact urticaria, urticaria due to cold and heat, cholinergic urticaria, other and unspecified urticaria.
  ② Outcomes: ADHD, BD, major depressive disorder (MDD), and SCZ.
2. Exploring the causal effect analysis of 91 inflammatory cytokines on 4 mental disorders (Figure 1: Step 2).
3. Explore the mediation analysis of inflammatory cytokines in the causal association of urticaria to mental disorders (Figure 1: Step 3).

**FIGURE 1:** A brief explanation of the design of the Mendelian Randomization (MR) model. Step 1 represents the MR research process of urticaria and mental disorders, which is the main analysis of this study; Step 2 represents the MR study process of inflammatory cytokines and selected mental disorders; In Step 3, c represents the process of Step 1, b represents the process of Step 2, and a represents the MR analysis process between urticaria and inflammatory cytokines. If there are significant differences in the results of processes a, b, and c, it indicates that inflammatory cytokines can mediate the pathway of urticaria to mental disorders. The image is created by Figdraw.

### 2.2 Instruments selection

Our study was based on three core assumptions of MR, namely (1) genetic IVs are highly correlated with exposure^16^; (2) genetic IVs are independent of confounders^22^; and (3) the only pathway leading to genetic variation is through exposure and not through any other pathway.^24^ To fulfil the above assumptions, we chose premium ideal IVs to guarantee the precision and comprehensiveness of the research findings. At first, when we tried to apply the commonly used significance threshold of *p* < 5 × 10^−8^, some of the exposed GWAS raw results had fewer significant loci, and after clumping pruning, the remaining valid IVs might only be in the single digits, which would lead to low statistical efficacy and weak IVs if MR analyses were performed, biasing the parameter estimates.^25^, ^26^ That is, when screening valid IVs for urticaria with its subtypes, we extracted SNPs at a relatively loose significance threshold of *p* < 5×10^−6^ (or *p* < 5× 10^−5^) and excluded SNPs with palindromic structures. In screening for effective IVs for inflammatory cytokines, we similarly extracted SNPs under the looser threshold of *p* < 5× 10^−6^ to increase the number of IVs available for each inflammatory cytokine. Furthermore, we used Steiger filtering^27^ to avoid the interference of reverse causal correlations as well as applied the following formula to calculate the *F*‐statistic with ensuring that the *F*‐statistic of the included SNPs were > 10 to exclude the influence of weak IVs on the results.^28^, ^29^

$$F=\frac{R^{2}\times \left(N-2\right)}{1-R^{2}}$$

where *N* denotes the sample size of the exposure (urticaria or inflammatory cytokines), *R* ^2^ denotes the proportion of exposures that can be explained for as IVs, which is usually calculated by the following equation:

$$R^{2}=\frac{\left[2\times \left(1-\mathrm{EAF}\right)\times \mathrm{EAF}\times \beta^{2}\right]}{\left[2\times \left(1-\mathrm{EAF}\right)\times \mathrm{EAF}\times \beta^{2}\right]+\left[2\times \mathrm{EAF}\times \left(1-\mathrm{EAF}\right)\times N\times \mathrm{SE}\left(\beta^{2}\right)\right]}$$

In the formula, *β* denotes the allele effect value, EAF denotes the frequency of the effect allele,^17^ and SE (*β*) denotes the standard error of genetic effect.^30^

Finally, IVs of urticaria and its subtypes were clustered within a 10 Mb genetic window using a strict linkage disequilibrium (LD) threshold of *r* ^2^ = 0.01. Additionally, IVs of inflammatory cytokines were clustered within a 10 Mb genetic window using an LD threshold of *r* ^2^ = 0.001. These screening conditions above set the correlation, independence, and statistical strength of the SNPs.

### 2.3 Data sources

The FinnGen study was a large‐scale genomics initiative that aimed to explore illness processes and susceptibility by correlating genetic variation with health data.^31^ The GWAS summary statistics for the urticaria and its subtypes were taken from version R10 published by the FinnGen Consortium (r10.finngen.fi), and all cases were diagnosed according to the International Classification of Diseases (ICD) codes ICD9 and ICD10 for a total of 398 204 patients with urticaria and its subtypes. A summary of the dataset, clinical diagnostic criteria, and other information about each subtype were available in Table S1. Basic information about the datasets can be found in Table 1, and all dataset populations were of European descent.

**TABLE 1:** Details of the GWAS included in the Mendelian randomization.

Diseases		GWAS ID/PubMed ID	Author	Year	Population	Sample size (*n* case vs. *n* control)	Consortium	Significance threshold
Urticaria	Urticaria	L12_URTICARIA	NA	2023	European	409 391 (11 187 vs. 398 204)	FinnGen	*p * < 5e‐6
	Allergic urticaria	L12_URTICA_ALLERG	NA	2023	European	400 823 (2619 vs. 398 204)	FinnGen	*p * < 5e‐6
	Dermatographic urticaria	L12_URTICA_DERTMATOG	NA	2023	European	400 282 (2078 vs. 398 204)	FinnGen	*p * < 5e‐6
	Contact urticaria	L12_URTIGA_CONTACT	NA	2023	European	398 292 (88 vs. 398 204)	FinnGen	*p * < 5e‐5
	Idiopathic urticaria	L12_URTICA_IDIOPAT	NA	2023	European	398 763 (559 vs. 398 204)	FinnGen	*p * < 5e‐5
	Urticaria due to cold and heat	L12_URTICA_COLDHEAT	NA	2023	European	398 438 (234 vs. 398 204)	FinnGen	*p * < 5e‐5
	Cholinergic urticaria	L12_URTICA_CHOLINERG	NA	2023	European	398 351 (147 vs. 398 204)	FinnGen	*p * < 5e‐5
	Other and unspecified urticaria	L12_URTICA_NAS	NA	2023	European	405 190 (6986 vs. 398 204)	FinnGen	*p * < 5e‐6
Inflammatory cytokines	91 Circulating inflammatory proteins	37563310	Jing Hua Zhao	2023	European	14 824	SCALLOP	*p* < 5e‐6
Mental disorders	ADHD	36702997	Ditte Demontis	2023	European	225 534 (38 691 vs. 186 843)	PGC	NA
	BD	34002096	Niamh Mullins	2021	European	413 466 (41 917 vs. 371 549)	PGC	NA
	MDD	30718901	David M. Howard	2019	European	500 199 (170 756 vs. 329 443)	PGC	NA
	SCZ	35396580	Vassily Trubetskoy	2022	European	130 644 (53 386 vs. 77 258)	PGC	NA

The specific information of 91 inflammatory cytokines is shown in Table S2. ADHD, attention deficit hyperactivity disorder; BD, bipolar disorder; GWAS, Genome Wide Association Study; MDD, major depressive disorder; NA, not available; PGC, Psychiatric Genomics Cooperation; SCALLOP, Systematic and Combined Analysis of Olink Proteins; SCZ, schizophrenia.

The greatest consortium and one of the most creative experiments in psychiatry's history is the Psychiatric Genomics Cooperation (PGC). The most significant meta‐ and mega‐analyses of genome‐wide genetic data on mental disorders have been carried out by it. The largest GWAS summary statistics on ADHD (38 691 cases and 186 843 controls),^32^ BD (41 917 cases and 371 549 controls),^33^ MDD (170 756 cases and 329 443 controls),^34^ and SCZ (53 386 cases and 77 258 controls)^35^ were extracted from the PGC (https://www.med.unc.edu/pgc/results‐and‐downloads/). In addition, data analyses, clinical diagnoses, and other information on each mental disorder can be found in Table S1. Detailed dataset information can be found in Table 1, with all samples from European pedigrees.

Summary‐level GWAS data on inflammatory cytokines were obtained from a recent study sponsored by the SCALLOP Consortium.^36^ The study recruited 11 cohorts for protein quantitative trait locus (pQTL) mapping by measuring 91 circulating inflammatory proteins using the Olink Targeted Inflammation Panel in 14 824 European participants, and performed a GWAS analysis for each protein in the pQTL mapping. Complete GWAS summary statistics for each inflammatory cytokines were available directly in the EBI GWAS Catalog (https://www.ebi.ac.uk/gwas/, accession numbers GCST90274758 to GCST90274848), and detailed information on each of the 91 inflammatory cytokines were available in Table S2.

### 2.4 Mendelian randomization and sensitivity analysis

To explore the association between urticaria and mental disorders, we conducted a two‐sample MR study mainly using the inverse variance weighting (IVW) method^37^ and selecting a random‐effects model. This method is by far the most important in MR analyses and has the advantage that in the absence of pleiotropy (and assuming that the selected IVs were valid), IVW tests for causal effects are unbiased.^38^, ^39^ To avoid bias in the IVW results due to uncertainty in the weak effects and level pleiotropy, we also introduced a novel Bayesian weighted Mendelian randomization (BWMR) approach to exclude chance bias due to horizontal pleiotropy.^40^, ^41^ The method infers a posteriori means of causal effects by means of the Variation Expectation Maximization (VEM) algorithm and adaptively detects outliers caused by pleiotropy.^41^ We considered the results valid when both the IVW and BWMR methods reached significant differences. In addition, MR‐egger, weighted median, weighted mode, and simple mode methods were further employed to verify the reliability of the causal relationship between exposure and outcome.

Finally, a sensitivity analysis was conducted to assess the possibility of violating the three core assumptions during MR. For the IVW approach, the MR‐PRESSO test was used to exclude outliers and reduce pleiotropy,^42^ followed by leave‐one‐out analyses to examine the effect of excluding selected individual SNP one by one on the overall results.^43^ Once an abnormal SNP was identified, we re‐ran the MR analysis after exclusion until no outliers were present. Cochran's Q test and funnel plots were used to test for heterogeneity among the included SNPs,^44^ and MR‐egger intercepts and their slope coefficients were used to validate horizontal pleiotropy of individual causal effects, which was represented as observed when *p*_intercept _< 0.05.^45^ In summary, sensitivity analyses were essential for analyzing potential heterogeneity and horizontal pleiotropy.

Odds ratios (ORs) and 95% confidence intervals (CIs) were used to determine the degree of binary causality. Multiple tests using the Bonferroni correction were defined as statistically significant when *p* < 0.0125 (*p* < 0.05/4) and were considered to imply the presence of nominal significance when 0.0125 <p< 0.05. All MR portions of the study followed the STROBE‐MR guidelines^46^ and were statistically analyzed using the TwoSampleMR (version 0.5.6) and MRPRESSO (version 1.0) software package in R (version 4.3.1, www.rproject.org/). For MR results scatter plots, leave‐one‐out analysis plots and forest plots can be found in the Supplementary figure.

## 3 RESULTS

### 3.1 Assessment of genetic IVs

Table 1 has shown participant‐specific characteristics from the FinnGen, GWAS Catalog, and PGC databases, including GWAS ID (or PubMed ID), author, year of publication, population characteristics, sample size, consortium for exposures and outcomes, as well as selected significance thresholds. After screening, specific information on all SNPs included in this study were provided in Tables S9–S11. The *F*‐statistics of all SNPs we selected in the three parts of MR study were > 16, suggesting that the effect of weak IVs on the results were almost negligible.

#### 3.1.1 Step 1: MR analysis results of urticaria on mental disorders

Figure 2 shows the results of a causal association between urticaria (and its seven subtypes) and four mental disorders in the MR analysis. After Bonferroni correction, our results revealed a range of significant and nominal associations. The results of IVW and BWMR together indicated a significant positive correlation between urticaria and the risk of developing ADHD (IVW: OR = 1.088, 95% CI: 1.026–1.154, *p* = 0.0051; BWMR: OR = 1.092, 95% CI: 1.025–1.163, *p* = 0.0064; Figure S1); a possible positive correlation between cholinergic urticaria and the risk of developing BD (IVW: OR = 1.012, 95% CI: 1.001–1.022, *p* = 0.0274; BWMR: OR = 1.013, 95% CI: 1.002–1.024, *p* = 0.025; Figure S10); a nominal positive correlation between dermatographic urticaria and the risk of developing ADHD (IVW: OR = 1.057, 95% CI: 1.005–1.112, *p* = 0.0323; BWMR: OR = 1.063, 95% CI: 1.007–1.122, *p* = 0.0276; Figure S17); a significant positive correlation between idiopathic urticaria and the risk of developing SCZ (IVW: OR = 1.013, 95% CI: 1.004–1.022, *p* = 0.0043; BWMR: OR = 1.013, 95% CI: 1.003–1.024, *p* = 0.0095; Figure S24); finally, a significant positive association between other unspecified urticaria and the risk of developing ADHD (IVW: OR = 1.085, 95% CI: 1.023–1.151, *p* = 0.0063; BWMR: OR = 1.09, 95% CI: 1.026–1.157, *p* = 0.0052; Figure S29). In addition, the results of IVW and BWMR were inconsistent between urticaria and the risk of developing MDD (IVW: *p* = 0.0497; BWMR: *p* = 0.0763; Figure S3), and also between idiopathic urticaria and the risk of developing MDD (IVW: *p* = 0.0346; BWMR: *p* = 0.0502; Figure S23), so we considered that these two results should be interpreted with caution. Finally, for allergic urticaria, urticaria due to cold and heat, and contact urticaria no evidence of association with the four mental disorders were found. The results of the five MR analysis methods for all urticaria (and its subtypes) in relation to mental disorders can be found in Table S3.

**FIGURE 2:** The main results of MR analysis on the causal relationship between urticaria and mental disorders (Step 1). Only results with significant differences are included, and detailed results can be obtained in Tables S3, S4. ADHD, attention deficit hyperactivity disorder; BD, bipolar disorder; BWMR, Bayesian weighted Mendelian randomization; CI, confidence interval; IVW, inverse‐variance weighted; MDD, major depressive disorder; MR, Mendelian randomization; OR, odds ratio; SCZ, schizophrenia; SNP, single‐nucleotide polymorphism.

To ensure the robustness of the resultant estimates, we need to validate our results through sensitivity analyses. The results of the sensitivity analyses were shown in Table S4, where the results of the Cochran'Q‐test showed that all *p*‐values > 0.05 and the funnel plots of all results were roughly symmetrical (Figures S1–S32), therefore no heterogeneity exists. The results of the MR‐Egger regression suggested a potential horizontal pleiotropy of idiopathic urticaria on ADHD (*p*_intercept_ = 0.014), despite our validation and exclusion efforts. In addition to this, the results of MR‐PRESSO did not reveal outliers in our analyses, and the leave‐one‐out method confirmed that deletion of a single IV did not affect the results.

#### 3.1.2 Step 2: MR analysis results of inflammatory cytokines on mental disorders

In this section, causal associations between 91 inflammatory cytokines and mental disorders (ADHD, BD, MDD, and SCZ) were explored, and significantly different results are shown in Figure 3, with detailed results available in Table S5. All results were co‐analyzed by IVW and BWMR methods. A total of six inflammatory cytokines were associated with ADHD, of which AXIN1 (IVW: OR = 1.141, 95% CI: 1.004–1.297, *p* = 0.044; Figure S33), CCL11 (IVW: OR = 1.07, 95% CI: 1.008–1.136, *p* = 0.025; Figure S34), FGF‐19 (IVW: OR = 1.077, 95% CI: 1.009–1.148, *p* = 0.025; Figure S36), and hGDNF (IVW: OR = 1.084, 95% CI: 1.014–1.159, *p* = 0.019; Figure S37) were risk factors for ADHD, whereas CD40 (IVW: OR = 0.933, 95% CI: 0.893–0.975, *p* = 0.002; Figure S35) and NT‐3 (IVW: OR = 0.875, 95% CI: 0.782–0.979, *p* = 0.019; Figure S38) were protective against ADHD.

**FIGURE 3:** The main results of MR analysis on the causal relationship between inflammatory cytokines and mental disorders (Step 2). ADHD, attention deficit hyperactivity disorder; BD, bipolar disorder; BWMR, Bayesian weighted Mendelian randomization; CI, confidence interval; IVW, inverse‐variance weighted; MDD, major depressive disorder; MR, Mendelian randomization; OR, odds ratio; SCZ, schizophrenia; SNP, single‐nucleotide polymorphism.

A total of six inflammatory cytokines were associated with BD. Among them, CXCL1 (IVW: OR = 1.066, 95% CI: 1.003–1.133, *p* = 0.041; Figure S39), FGF‐5 (IVW: OR = 1.048, 95% CI: 1.005–1.093, *p* = 0.027; Figure S41), and hGDNF (IVW: OR = 1.094, 95% CI: 1.023–1.171, *p* = 0.009; Figure S42) were risk factors for BD, while CXCL5 (IVW: OR = 0.944, 95% CI: 0.901–0.99, *p* = 0.018; Figure S40), HGF (IVW: OR = 0.879, 95% CI: 0.792–0.976, *p* = 0.016; Figure S43), and IL‐20 (IVW: OR = 0.900, 95% CI: 0.813–0.995, *p* = 0.040; Figure S44) were protective against BD.

A total of four inflammatory cytokines were associated with MDD, of which CCL19 (IVW: OR = 1.036, 95% CI: 1.001–1.072, *p* = 0.045; Figure S45), IFN‐γ (IVW: OR = 1.053, 95% CI: 1.001–1.108, *p* = 0.046; Figure S46), and TGF‐α (IVW: OR = 1.075, 95% CI: 1.015–1.138, *p* = 0.014; Figure S47) were risk factors for MDD, whereas TNFB (IVW: OR = 0.965, 95% CI: 0.934–0.996, *p* = 0.027; Figure S48) was protective against MDD.

Finally, for SCZ, there were inconsistent findings to explore the impact of IL‐24 on SCZ using IVW and BWMR methods (IVW: *p* = 0.041; BWMR: *p* = 0.051; Figure S53), so the results should be interpreted with caution. In addition to this, a total of four cytokines were causally associated with SCZ. Among them, 4EBP1 (IVW: OR = 1.099, 95% CI: 1.006–1.201, *p* = 0.036; Figure S49) and DNER (IVW: OR = 1.118, 95% CI: 1.058–1.182, *p* <0.001; Figure S51) were risk factor for SCZ, while CD40 (IVW: OR = 0.92, 95% CI: 0.873–0.969, *p* = 0.002; Figure S50) and IL‐5 (IVW: OR = 0.903, 95% CI: 0.828–0.983, *p* = 0.019; Figure S52) were protective factor for SCZ.

We verified the results of this section by sensitivity analysis and did not find potential heterogeneity (Cochran's Q *p* > 0.05). In addition, both MR‐PRESSO and MR‐Egger regression did not reveal outliers or horizontal pleiotropy in our analyses, and the leave‐one‐out method confirmed that the results were robust (Table S6).

#### 3.1.3 Step 3: Mediation analysis

After Steps 1 and 2, both urticaria and inflammatory cytokines were causally associated with mental disorders. Inflammatory cytokines might have mediated the pathway between urticaria and mental disorders. Therefore, one of the validation methods was that urticaria was also significantly correlated with inflammatory cytokines (Step 3a in Figure 1). However, this portion of the results indicated that there was no causal relationship between urticaria associated with mental disorders and inflammatory cytokines associated with mental disorders (Tables S7, S8 and Figures S54–S70). In other words, inflammatory cytokines did not mediate the pathway by which urticaria led to mental disorders.

## 4 DISCUSSION

In this study, MR analysis was used for the first time to verify the causal relationship between urticaria and four common mental disorders. IVW and BWMR methods together revealed that urticaria was significantly associated with an increased risk of developing ADHD. Among the urticaria subtypes, cholinergic urticaria significantly increased the risk of BD; dermatographic urticaria may be associated with an increased risk of ADHD; idiopathic urticaria significantly increased the risk of SCZ; and other unspecified urticaria was significantly associated with an increased risk of ADHD. We also explored whether inflammatory cytokines act as mediators to mediate the process of urticaria and mental disorders by MR methods. The results indicated that eight inflammatory cytokines were negatively associated with selected mental disorders and 12 inflammatory factors were positively associated with mental disorders, but they did not act as a mediator between urticaria and mental disorders.

Many dermatologic disorders are now thought to be potentially related to mental disorders. For example, atopic dermatitis have been found to be associated with an increased prevalence of anxiety and depression in adults,^47^ which was subsequently validated in an MR study.^48^ Subsequently, a study pooled 14 GWAS summary‐level datasets and used MR methods to confirm that negative emotions (depression, guilt, mood swings, etc.) all correlate with psoriasis.^49^ In addition, observational studies have found an increased risk of depression and anxiety in patients with acne,^50^, ^51^ and alopecia areata also leads to an increased risk of major depression.^52^ And urticaria, a typical allergic skin disease, is also thought to be associated with an increased risk of developing mental disorders. A population‐based study found that CU patients had a higher probability of developing mental disorders, of which somatic disorder and depression were the most prevalent mental disorders.^53^ Another meta‐analysis based on 25 studies found that nearly one‐third of CU patients had at least one underlying mental disorder.^54^ Tat ^55^ also found that sleep‐wake disorders were also highly common in CU patients. Our study also found a causal association between urticaria (including dermatographic urticaria, other and unspecified urticaria) and an increased risk of developing ADHD. In fact, Chen et al.^56^ found a higher prevalence of ADHD in patients with urticaria than in controls, whereas ADHD did not increase the prevalence of urticaria in a two‐sample MR study,^57^ suggested that the increased incidence of ADHD due to urticaria is not disturbed by reverse causality. Additionally, this study also found that cholinergic urticaria might have increased the risk of BD, and idiopathic urticaria could have raised the risk of SCZ. In fact, there were very few studies on the association between urticaria and BD or SCZ. A Danish population‐based study found that hospital contact with any atopic disease increased the risk of SCZ by 1.45 times, but this significant increase in risk was only observed when atopic dermatitis, urticaria, and allergic rhinitis were combined into one group.^58^ Another study that investigated the general medical conditions (GMC) of BD patients found that urticaria was one of the most commonly reported GMCs, suggesting a potential link between BD and urticaria.^59^ In our study, almost all confounding factors affecting the results were reduced, resulting in more reliable evidence and more credible conclusions.

This study confirms the causal link between urticaria and mental disorders, indicating that enhancing the mental health of individuals with urticaria could help alleviate the current burden of mental disorders in society. This finding implies that reducing the frequency of urticaria episodes might lead to improvements in psychiatric issues. For instance, Gupta^60^ and Hashiro^61^ concurrently treated patients with antiallergics, psychotropic medications (such as antidepressants and benzodiazepines), and psychotherapy, suggesting that this approach could have been beneficial in managing urticaria and curbing the progression of mental disorders. Further research is needed to solidify this connection in the future.

The pathophysiological mechanism between urticaria and mental disorders is currently uncertain.^62^, ^63^, ^64^ A seemingly plausible explanation at present assumes that the interaction between urticaria and the CNS may be mediated by the immune system.^11^, ^12^ The basis of mental disorders and the pathogenesis of many allergic skin diseases may be the “brain‐skin” connection of local neuro‐immune‐endocrine circuits.^65^, ^66^, ^67^ There seems to be a pathway to explain how inflammatory dysregulation affects brain changes. For example, peripheral inflammatory markers can affect the brain directly and without crossing the BBB at all.^54^ Inflammatory responses may also increase the permeability of the BBB, making the brain susceptible to inflammatory cytokines and autoantibodies, which can trigger neurological symptoms when exposed to the brain.^68^, ^69^, ^70^ Urticaria typically causes elevated levels of pro‐inflammatory cytokines, and increases in cytokines may lead to depression, anxiety, and autism.^71^ A systematic review suggested that sustained excessive release of inflammatory mediators from the atopic response may affect brain circuits associated with ADHD, with children being the most susceptible to ADHD symptoms.^72^ Thus, inflammatory cytokines may serve as an important link between urticaria and mental disorders. We continued to use MR methods to explore causal associations between inflammatory cytokines and mental disorders (step 2). The results indicated that some inflammatory cytokines were causally related to mental disorders as follows: For ADHD, AXIN1, CCL11, FGF‐19, and hGDNF were risk factors for ADHD, whereas CD40 and NT‐3 were protective against ADHD. For BD, CXCL1, FGF‐5, and hGDNF were risk factors for BD, whereas CXCL5, HGF, and IL‐20 were protective against BD. For MDD, CCL19, IFN‐γ, and TGF‐α were risk factors for MDD, whereas TNFB was protective against MDD. Finally, for SCZ, 4EBP1 and DNER were risk factors for SCZ, whereas CD40 and IL‐5 were protective factors for SCZ. A study suggested that bidirectional communication between neurons and immune cells may exist and can cooperate to regulate synaptic plasticity and neuroimmunity.^73^ Cytokines can cross the BBB via periventricular organs and specific transport proteins. After brain injury,^74^ the CNS activates microglia and initiates complex neuroinflammatory signaling pathways that produce and release a wider variety of cytokines that can lead to persistent neuroinflammation associated with a variety of neurological disorders.^75^ And stress‐related activation of microglia in a prolonged pro‐inflammatory state may be directly related to depressive behaviors and anxiety.^76^ IL‐23, IL‐6, IL‐1β, IFN‐γ, TNF, and GM‐CSF are usually the key factors associated with neuroinflammation, of which IL‐1β and IL‐6 are the two most relevant cytokines for mental disorders in the inflamed CNS.^77^, ^78^ In present study, we did not find any mental disorders associated with IL‐1β or IL‐6, but we confirmed a causal association of IFN‐γ with an increased risk of developing MDD. Several studies have demonstrated that patients with MDD had significantly higher serum levels of IFN‐γ than controls.^79^, ^80^, ^81^ And the higher the IFN‐γ level, the poorer the sleep quality of MDD patients.^80^ IFN‐γ is often thought to be associated with an abnormal neuroinflammatory response, including hyperactivation of microglia and recruitment of other immune cells.^82^ Therefore, IFN‐γ is also expected to be a co‐diagnostic factor for MDD.^79^ In addition to IFN‐γ, higher levels of human Glial cell line‐derived neurotrophic factor (hGDNF) has been demonstrated to be associated with ADHD.^83^, ^84^ hGDNF is considered a type of neurotrophic factors (NTs), which is also involved in promoting neuronal growth, survival, and differentiation and is highly expressed in the striatum.^85^ It interacts with glutamate to regulate neuronal development, and dysregulation may alter glutamate signaling, which may lead to symptoms of mental disorders.^86^ Our findings also provided new evidence that hGDNF causes an increased risk of ADHD, hence previous studies were considered reliable.

Next, we performed MR analysis of urticaria and inflammatory cytokines, which once an association between the two was confirmed, could indicate that inflammatory cytokines could act as mediators to mediate urticaria‐induced mental disorders. However, the final results showed no causal association between urticaria and inflammatory cytokines related to mental disorders. In other words, inflammatory cytokines may not be the pathway that mediates urticaria‐induced mental disorders. This is inconsistent with the results of many previous studies. We believe that there are many reasons for the inconsistent results. First of all, the effects of urticaria on the brain may also be related to its effects on the neurotransmitter system.^87^ Studies have shown that urticaria may lead to abnormal increases in neurotransmitters (such as dopamine, glutamate, and gamma‐aminobutyric acid), affecting the normal functioning of the brain.^87^, ^88^, ^89^ These changes may increase the incidence of mental disorders such as ADHD, SCZ, and BD. Second, previous studies may have been potentially influenced by confounding factors, including self‐reported urticaria, the way outcomes were measured and defined, selection bias across samples, and varying degrees of other external factors (age, gender, and comorbidities) that may have confounded pathogenesis.^90^ Finally, even though we chose the most current GWAS statistics for 91 inflammatory factors, there are still more neural‐related inflammatory cytokines that were not included, and thus the interpretation of the results of this part of our study (Step 3) is limited.

The key strength of this study is mainly the design of the MR methodology, where we divided the analysis into three parts, utilizing two‐sample MR at each step, and once the presence of the mediator is confirmed, we calculate the mediating effect. In addition, we introduced the latest MR analysis method, the BWMR approach, which is computationally stable and statistically valid compared to existing correlation methods. For the selection of databases, we all chose the latest and largest GWAS database in order to maximize the validation of our hypotheses. However, this study still has some limitations. First, the populations in the GWAS database are of European origin, and there is no current GWAS statistical database for urticaria or mental disorders that is categorized by sex or age, so the present study may be biased in terms of population stratification. Second, the influence of the Beavis effect (or winner's curse) still cannot be ruled out in MR studies,^91^ but the bias was minimized as much as possible by rigorous screening and statistical methods. Finally, there may be differences between MR and observational studies or randomized controlled trials, whose estimates are usually larger than those of observational studies,^92^ thus requiring more caution in interpreting results estimated from different studies.

## 5 CONCLUSIONS

In conclusion, we comprehensively explored the genetic causality between urticaria, inflammatory cytokines, and mental disorders. The results showed that urticaria and its subtypes were significantly associated with an increased risk of developing four common mental disorders. Next, we found that eight inflammatory cytokines were negatively associated with selected mental disorders and 12 inflammatory factors were positively associated with mental disorders. Finally, our findings suggest that inflammatory cytokines do not act as mediators to influence the pathway between urticaria and mental disorders. We suggest that the treatment of urticaria could appropriately incorporate psychiatric interventions (pharmacologic or psychological) and timely mental health assessment of patients with urticaria, and that collaboration between dermatologists and psychiatrists is also expected to improve patients’ symptoms and quality of life. In addition, we hope that smaller deviant MR methods or larger combined GWAS datasets will be developed in the future to validate or update our findings with new studies.

## DECLARATIONS

This study only used published and publicly available data. Ethical approval for each study included in the investigation can be found in the original publications (including informed consent from each participant).

## CONFLICT OF INTEREST STATEMENT

The authors declare no competing interests.

## Supporting information

Supporting Information

Supporting Information

Supporting Information

Supporting Information

Supporting Information

Supporting Information

Supporting Information

## Data Availability

All original data are available at the following URL: 1. https://pgc.unc.edu/for‐researchers/download‐results/, 2. https://r10.finngen.fi/, 3. https://www.finngen.fi/en/access_results, 4. https://www.ebi.ac.uk/gwas/.

## References

[1] Kolkhir P , Giménez‐Arnau A , Kulthanan K , Peter J , Metz M , Maurer M . Urticaria. Nat Rev Dis Primers. 2022;8(1):61. 10.1038/s41572-022-00389-z 36109590

[2] Krause K , Grattan C , Bindslev‐Jensen C , et al. How not to miss autoinflammatory diseases masquerading as urticaria. Allergy. 2012;67(12):1465‐1474. 10.1111/all.12030 22978406

[3] Radonjic‐Hoesli S , Hofmeier K , Micaletto S , Schmid‐Grendelmeier P , Bircher A , Simon D . Urticaria and angioedema: an update on classification and pathogenesis. Clin Rev Allergy Immunol. 2018;54(1):88‐101. 10.1007/s12016-017-8628-1 28748365

[4] Zuberbier T , Abdul LA , Abuzakouk M , et al. The international EAACI/GA^2^LEN/EuroGuiDerm/APAAACI guideline for the definition, classification, diagnosis, and management of urticaria. Allergy. 2022;77(3):734‐766. 10.1111/all.15090 34536239

[5] Greaves M . Autoimmune urticaria. Clin Rev Allergy Immunol. 2002;23(2):171‐183. 10.1385/criai:23:2:171 12221862

[6] Lang D . Chronic urticaria. N Engl J Med. 2022;387(9):824‐831. 10.1056/NEJMra2120166 36053507

[7] Altınöz A , Taşkıntuna N , Altınöz S , Ceran S . A cohort study of the relationship between anger and chronic spontaneous urticaria. Adv Ther. 2014;31(9):1000‐1007. 10.1007/s12325-014-0152-6 25209876

[8] O'Donnell B , Lawlor F , Simpson J , Morgan M , Greaves M . The impact of chronic urticaria on the quality of life. Br J Dermatol. 1997;136(2):197‐201.9068731

[9] Potocka A , Turczyn‐Jabloñska K , Merecz D . Psychological correlates of quality of life in dermatology patients: the role of mental health and self‐acceptance. Acta Dermatovenerol Alp Pannonica Adriat. 2009;18(2):53‐58, 60, 62.19588058

[10] Choi G , Nam Y , Park C , et al. Anxiety, depression, and stress in Korean patients with chronic urticaria. Korean J Intern Med. 2020;35(6):1507‐1516. 10.3904/kjim.2019.320 32450676 PMC7652653

[11] Paus R , Theoharides T , Arck P . Neuroimmunoendocrine circuitry of the ‘brain‐skin connection’. Trends Immunol. 2006;27(1):32‐39. 10.1016/j.it.2005.10.002 16269267

[12] Segerstrom S , Miller G . Psychological stress and the human immune system: a meta‐analytic study of 30 years of inquiry. Psychol Bull. 2004;130(4):601‐630. 10.1037/0033-2909.130.4.601 15250815 PMC1361287

[13] Weller K , Koti I , Makris M , Maurer M . Anxiety and depression seem less common in patients with autoreactive chronic spontaneous urticaria. Clin Exp Dermatol. 2013;38(8):870‐873. 10.1111/ced.12190 23889120

[14] Oguz Topal I , Kıvanc Altunay I , Mercan S . Personality disorders, anxiety and depression in the patients with chronic urticaria. Turkish J Clin Psy. 2004;7(4):199‐209.

[15] Sheehan‐Dare R , Henderson M , Cotterill J . Anxiety and depression in patients with chronic urticaria and generalized pruritus. Br J Dermatol. 1990;123(6):769‐774. 10.1111/j.1365-2133.1990.tb04195.x 2265093

[16] Smith G , Ebrahim S . ‘Mendelian randomization’: can genetic epidemiology contribute to understanding environmental determinants of disease? Int J Epidemiol. 2003;32(1):1‐22. 10.1093/ije/dyg070 12689998

[17] Davey SG , Hemani G . Mendelian randomization: genetic anchors for causal inference in epidemiological studies. Hum Mol Genet. 2014;23(R1):R89‐R98. 10.1093/hmg/ddu328 25064373 PMC4170722

[18] Evans D , Davey SG . Mendelian randomization: new applications in the coming age of hypothesis‐free causality. Annu Rev Genomics Hum Genet. 2015;16:327‐350. 10.1146/annurev-genom-090314-050016 25939054

[19] Lawlor D , Harbord R , Sterne J , Timpson N , Davey SG . Mendelian randomization: using genes as instruments for making causal inferences in epidemiology. Stat Med. 2008;27(8):1133‐1163. 10.1002/sim.3034 17886233

[20] Burgess S , Small D , Thompson S . A review of instrumental variable estimators for Mendelian randomization. Stat Methods Med Res. 2017;26(5):2333‐2355. 10.1177/0962280215597579 26282889 PMC5642006

[21] Holmes M , Ala‐Korpela M , Smith G . Mendelian randomization in cardiometabolic disease: challenges in evaluating causality. Nat Rev Cardiol. 2017;14(10):577‐590. 10.1038/nrcardio.2017.78 28569269 PMC5600813

[22] Emdin C , Khera A , Kathiresan S . Mendelian randomization. JAMA. 2017;318(19):1925‐1926. 10.1001/jama.2017.17219 29164242

[23] Davies N , Holmes M , Davey SG . Reading Mendelian randomisation studies: a guide, glossary, and checklist for clinicians. BMJ. 2018;362:k601. 10.1136/bmj.k601 30002074 PMC6041728

[24] Smith G , Lawlor D , Harbord R , Timpson N , Day I , Ebrahim S . Clustered environments and randomized genes: a fundamental distinction between conventional and genetic epidemiology. PLoS Med. 2007;4(12):e352. 10.1371/journal.pmed.0040352 18076282 PMC2121108

[25] Lawlor D , Wade K , Borges M , et al. A Mendelian randomization dictionary: useful definitions and descriptions for undertaking, understanding and interpreting Mendelian randomization studies. OSF Preprints. 2019. 10.31219/osf.io/6yzs7

[26] Wang J , Zhang L . Correlation between cigarette smoking and alcohol consumption and Rosacea: a two‐sample Mendelian randomization study. Skin Res Technol. 2024;30(6):e13765. 10.1111/srt.13765 38881049 PMC11180680

[27] Hemani G , Tilling K , Davey Smith G . Orienting the causal relationship between imprecisely measured traits using GWAS summary data. PLoS Genet. 2017;13(11):e1007081. 10.1371/journal.pgen.1007081 29149188 PMC5711033

[28] Burgess S , Thompson S . Avoiding bias from weak instruments in Mendelian randomization studies. Int J Epidemiol. 2011;40(3):755‐764. 10.1093/ije/dyr036 21414999

[29] Palmer T , Lawlor D , Harbord R , et al. Using multiple genetic variants as instrumental variables for modifiable risk factors. Stat Methods Med Res. 2012;21(3):223‐242. 10.1177/0962280210394459 21216802 PMC3917707

[30] Shim H , Chasman D , Smith J , et al. A multivariate genome‐wide association analysis of 10 LDL subfractions, and their response to statin treatment, in 1868 Caucasians. PLoS ONE. 2015;10(4):e0120758. 10.1371/journal.pone.0120758 25898129 PMC4405269

[31] Kurki M , Karjalainen J , Palta P , et al. FinnGen provides genetic insights from a well‐phenotyped isolated population. Nature. 2023;613(7944):508‐518. 10.1038/s41586-022-05473-8 36653562 PMC9849126

[32] Demontis D , Walters G , Athanasiadis G , et al. Genome‐wide analyses of ADHD identify 27 risk loci, refine the genetic architecture and implicate several cognitive domains. Nat Genet. 2023;55(2):198‐208. 10.1038/s41588-022-01285-8 36702997 PMC10914347

[33] Mullins N , Forstner A , O'Connell K , et al. Genome‐wide association study of more than 40,000 bipolar disorder cases provides new insights into the underlying biology. Nat Genet. 2021;53(6):817‐829. 10.1038/s41588-021-00857-4 34002096 PMC8192451

[34] Howard D , Adams M , Clarke T , et al. Genome‐wide meta‐analysis of depression identifies 102 independent variants and highlights the importance of the prefrontal brain regions. Nat Neurosci. 2019;22(3):343‐352. 10.1038/s41593-018-0326-7 30718901 PMC6522363

[35] Trubetskoy V , Pardiñas A , Qi T , et al. Mapping genomic loci implicates genes and synaptic biology in schizophrenia. Nature. 2022;604(7906):502‐508. 10.1038/s41586-022-04434-5 35396580 PMC9392466

[36] Zhao JH , Stacey D , Eriksson N , et al. Genetics of circulating inflammatory proteins identifies drivers of immune‐mediated disease risk and therapeutic targets. Nat Immunol. 2023;24(9):1540‐1551. 10.1038/s41590-023-01588-w 37563310 PMC10457199

[37] Lee CH , Cook S , Lee JS , Han B . Comparison of two meta‐analysis methods: inverse‐variance‐weighted average and weighted sum of Z‐scores. Genomics Inform. 2016;14(4):173‐180. 10.5808/gi.2016.14.4.173 28154508 PMC5287121

[38] Hemani G , Zheng J , Elsworth B , et al. The MR‐base platform supports systematic causal inference across the human phenome. eLife. 2018;7:e34408. 10.7554/eLife.34408 29846171 PMC5976434

[39] Bowden J , Davey SG , Burgess S . Mendelian randomization with invalid instruments: effect estimation and bias detection through Egger regression. Int J Epidemiol. 2015;44(2):512‐525. 10.1093/ije/dyv080 26050253 PMC4469799

[40] Zhao J , Ming J , Hu X , Chen G , Liu J , Yang C . Bayesian weighted Mendelian randomization for causal inference based on summary statistics. Bioinformatics. 2020;36(5):1501‐1508. 10.1093/bioinformatics/btz749 31593215

[41] Grant A , Burgess S . A Bayesian approach to Mendelian randomization using summary statistics in the univariable and multivariable settings with correlated pleiotropy. Am J Hum Genet. 2024;111(1):165‐180. 10.1016/j.ajhg.2023.12.002 38181732 PMC10806746

[42] Verbanck M , Chen CY , Neale B , Do R . Detection of widespread horizontal pleiotropy in causal relationships inferred from Mendelian randomization between complex traits and diseases. Nat Genet. 2018;50(5):693‐698. 10.1038/s41588-018-0099-7 29686387 PMC6083837

[43] Gu X , Guo T , Si Y , et al. Association between ambient air pollution and daily hospital admissions for depression in 75 Chinese cities. Am J Psychiatry. 2020;177(8):735‐743. 10.1176/appi.ajp.2020.19070748 32312109

[44] Cohen J , Chalumeau M , Cohen R , Korevaar D , Khoshnood B , Bossuyt P . Cochran's Q test was useful to assess heterogeneity in likelihood ratios in studies of diagnostic accuracy. J Clin Epidemiol. 2015;68(3):299‐306. 10.1016/j.jclinepi.2014.09.005 25441698

[45] Burgess S , Thompson S . Interpreting findings from Mendelian randomization using the MR‐Egger method. Eur J Epidemiol. 2017;32(5):377‐389. 10.1007/s10654-017-0255-x 28527048 PMC5506233

[46] Skrivankova VW , Richmond RC , Woolf BAR , et al. Strengthening the reporting of observational studies in epidemiology using Mendelian randomization: the STROBE‐MR statement. JAMA. 2021;326(16):1614‐1621. 10.1001/jama.2021.18236 34698778

[47] Henderson A , Adesanya E , Mulick A , et al. Common mental health disorders in adults with inflammatory skin conditions: nationwide population‐based matched cohort studies in the UK. BMC Med. 2023;21(1):285. 10.1186/s12916-023-02948-x 37542272 PMC10403838

[48] Chu M , Shen S , Zhu Z , et al. Association of psoriasis with depression, anxiety, and suicidality: a bidirectional two‐sample Mendelian randomization study. J Dermatol. 2023;50(12):1629‐1634. 10.1111/1346-8138.16941 37697936

[49] Zhang M , Hu Y , Chen L , et al. Roles of negative emotions and personality traits in psoriasis vulgaris: a Mendelian randomization study. Skin Res Technol. 2024;30(5):e13702. 10.1111/srt.13702 38743386 PMC11093070

[50] Samuels D , Rosenthal R , Lin R , Chaudhari S , Natsuaki M . Acne vulgaris and risk of depression and anxiety: a meta‐analytic review. J Am Acad Dermatol. 2020;83(2):532‐541. 10.1016/j.jaad.2020.02.040 32088269

[51] Vallerand I , Lewinson R , Parsons L , et al. Risk of depression among patients with acne in the U.K.: a population‐based cohort study. Br J Dermatol. 2018;178(3):e194‐e195. 10.1111/bjd.16099 29411352

[52] Yu N , Guo Y . Association between alopecia areata, anxiety, and depression: insights from a bidirectional two‐sample Mendelian randomization study. J Affect Disord. 2024;350:328‐331. 10.1016/j.jad.2024.01.152 38242214

[53] Chu C , Cho Y , Jiang J , Chang C , Liao S , Tang C . Patients with chronic urticaria have a higher risk of psychiatric disorders: a population‐based study. Br J Dermatol. 2020;182(2):335‐341. 10.1111/bjd.18240 31220338

[54] Konstantinou G , Konstantinou G . Psychiatric comorbidity in chronic urticaria patients: a systematic review and meta‐analysis. Clin Trans Allergy. 2019;9:42. 10.1186/s13601-019-0278-3 PMC670689431462988

[55] Tat T . Higher levels of depression and anxiety in patients with chronic urticaria. Med Sci Monit. 2019;25:115‐120. doi:10.12659/msm.912362 30609422 PMC6329254

[56] Chen M , Su T , Chen Y , et al. Comorbidity of allergic and autoimmune diseases among patients with ADHD. J Atten Disord. 2017;21(3):219‐227. 10.1177/1087054712474686 23400216

[57] Zhang X , Zhang R , Zhang Y , Lu T . Associations between attention‐deficit/hyperactivity disorder and allergic diseases: a two‐sample Mendelian randomization study. Front Psychiatry. 2023;14:1185088. 10.3389/fpsyt.2023.1185088 37484661 PMC10356558

[58] Pedersen M , Benros M , Agerbo E , Børglum A , Mortensen P . Schizophrenia in patients with atopic disorders with particular emphasis on asthma: a Danish population‐based study. Schizophr Res. 2012;138(1):58‐62. 10.1016/j.schres.2012.02.019 22391212

[59] Perugi G , Quaranta G , Belletti S , et al. General medical conditions in 347 bipolar disorder patients: clinical correlates of metabolic and autoimmune‐allergic diseases. J Affect Disord. 2015;170:95‐103. 10.1016/j.jad.2014.08.052 25237732

[60] Gupta M , Gupta A . Chronic idiopathic urticaria associated with panic disorder: a syndrome responsive to selective serotonin reuptake inhibitor antidepressants? Cutis. 1995;56(1):53‐54.7555104

[61] Hashiro M . Psychosomatic treatment of a case of chronic urticaria. J Dermatol. 1995;22(9):686‐689. 10.1111/j.1346-8138.1995.tb03899.x 8537557

[62] Caccavale S , Bove D , Bove R , La MM . Skin and brain: itch and psychiatric disorders. G Ital Dermatol Venereol. 2016;151(5):525‐529.25854671

[63] Consoli S . Psychological factors in chronic urticaria. Ann Dermatol Venereol. 2023;130 Spec No 1:1s73‐7.12843812

[64] Gregoriou S , Rigopoulos D , Katsambas A , et al. Etiologic aspects and prognostic factors of patients with chronic urticaria: nonrandomized, prospective, descriptive study. J Cutan Med Surg. 2009;13(4):198‐203. 10.2310/7750.2008.08035 19706227

[65] Dalman C , Allebeck P , Gunnell D , et al. Infections in the CNS during childhood and the risk of subsequent psychotic illness: a cohort study of more than one million Swedish subjects. Am J Psychiatry. 2008;165(1):59‐65. 10.1176/appi.ajp.2007.07050740 18056223

[66] Eaton W , Byrne M , Ewald H , et al. Association of schizophrenia and autoimmune diseases: linkage of Danish national registers. Am J Psychiatry. 2006;163(3):521‐528. 10.1176/appi.ajp.163.3.521 16513876

[67] Niebuhr D , Millikan A , Cowan D , Yolken R , Li Y , Weber N . Selected infectious agents and risk of schizophrenia among U.S. military personnel. Am J Psychiatry. 2008;165(1):99‐106. 10.1176/appi.ajp.2007.06081254 18086751

[68] Lennox B , Coles A , Vincent A . Antibody‐mediated encephalitis: a treatable cause of schizophrenia. Br J Psychiatry. 2012;200(2):92‐94. 10.1192/bjp.bp.111.095042 22297586

[69] Diamond B , Huerta P , Mina‐Osorio P , Kowal C , Volpe B . Losing your nerves? Maybe it's the antibodies. Nat Rev Immunol. 2009;9(6):449‐456. 10.1038/nri2529 19424277 PMC2783680

[70] Dantzer R , O'Connor J , Freund G , Johnson R , Kelley K . From inflammation to sickness and depression: when the immune system subjugates the brain. Nat Rev Neurosci. 2008;9(1):46‐56. 10.1038/nrn2297 18073775 PMC2919277

[71] Pollak Y , Yirmiya R . Cytokine‐induced changes in mood and behaviour: implications for ‘depression due to a general medical condition’, immunotherapy and antidepressive treatment. Int J Neuropsychopharmacol. 2002;5(4):389‐399. 10.1017/s1461145702003152 12466037

[72] Schmitt J , Buske‐Kirschbaum A , Roessner V . Is atopic disease a risk factor for attention‐deficit/hyperactivity disorder? A systematic review. Allergy. 2010;65(12):1506‐1524. 10.1111/j.1398-9995.2010.02449.x 20716320

[73] Almeida P , Nani J , Oses J , Brietzke E , Hayashi M . Neuroinflammation and glial cell activation in mental disorders. Brain Behav Immun Health. 2020;2:100034. 10.1016/j.bbih.2019.100034 38377429 PMC8474594

[74] Limanaqi F , Biagioni F , Gaglione A , Busceti C , Fornai F . A sentinel in the crosstalk between the nervous and immune system: the (immuno)‐proteasome. Front Immunol. 2019;10:628. 10.3389/fimmu.2019.00628 30984192 PMC6450179

[75] Carson M , Doose J , Melchior B , Schmid C , Ploix C . CNS immune privilege: hiding in plain sight. Immunol Rev. 2006;213:48‐65. 10.1111/j.1600-065X.2006.00441.x 16972896 PMC2633103

[76] Sun R , Zhao Z , Feng J , et al. Glucocorticoid‐potentiated spinal microglia activation contributes to preoperative anxiety‐induced postoperative hyperalgesia. Mol Neurobiol. 2017;54(6):4316‐4328. 10.1007/s12035-016-9976-1 27339881

[77] Hu W , Holtzman D , Fagan A , et al. Plasma multianalyte profiling in mild cognitive impairment and Alzheimer disease. Neurology. 2012;79(9):897‐905. 10.1212/WNL.0b013e318266fa70 22855860 PMC3425844

[78] Patel NS , Paris D , Mathura V , Quadros AN , Crawford FC , Mullan MJ . Inflammatory cytokine levels correlate with amyloid load in transgenic mouse models of Alzheimer's disease. J Neuroinflam. 2005;2(1):9. 10.1186/1742-2094-2-9 PMC55555715762998

[79] Chen S , Zhang Y , Yuan Y . The combination of serum BDNF, cortisol and IFN‐gamma can assist the diagnosis of major depressive disorder. Neuropsychiatr Dis Treat. 2021;17:2819‐2829. 10.2147/ndt.S322078 34471356 PMC8405229

[80] Yang Y , Gu K , Meng C , et al. Relationship between sleep and serum inflammatory factors in patients with major depressive disorder. Psychiatry Res. 2023;329:115528. 10.1016/j.psychres.2023.115528 37837811

[81] Lu L , Hu X , Jin X . IL‐4 as a potential biomarker for differentiating major depressive disorder from bipolar depression. Medicine (Baltimore). 2023;102(15):e33439. 10.1097/md.0000000000033439 37058046 PMC10101271

[82] Shi Y , Wei B , Li L , Wang B , Sun M . Th17 cells and inflammation in neurological disorders: possible mechanisms of action. Front Immunol. 2022;13:932152. 10.3389/fimmu.2022.932152 35935951 PMC9353135

[83] Bilgiç A , Toker A , Işık Ü , Kılınç İ. Serum brain‐derived neurotrophic factor, glial‐derived neurotrophic factor, nerve growth factor, and neurotrophin‐3 levels in children with attention‐deficit/hyperactivity disorder. Eur Child Adolesc Psychiatry. 2017;26(3):355‐363. 10.1007/s00787-016-0898-2 27561780

[84] Niitsu T , Oda Y , Idemoto K , et al. Association between serum levels of glial cell line‐derived neurotrophic factor and inattention in adult patients with attention deficits/hyperactivity disorder. Psychiatry Res. 2021;296:113674. 10.1016/j.psychres.2020.113674 33385784

[85] Huertas‐Fernández I , Gómez‐Garre P , Madruga‐Garrido M , et al. GDNF gene is associated with tourette syndrome in a family study. Mov Disord. 2015;30(8):1115‐1120. 10.1002/mds.26279 26096985 PMC5036394

[86] Mattson M . Glutamate and neurotrophic factors in neuronal plasticity and disease. Ann NY Acad Sci. 2008;1144:97‐112. 10.1196/annals.1418.005 19076369 PMC2614307

[87] Tomaszewska K , Słodka A , Tarkowski B , Zalewska‐Janowska A . Neuro‐immuno‐psychological aspects of chronic urticaria. J Clin Med. 2023;12(9):3134. 10.3390/jcm12093134 37176575 PMC10179371

[88] Pondeljak N , Lugović‐Mihić L . Stress‐induced interaction of skin immune cells, hormones, and neurotransmitters. Clin Ther. 2020;42(5):757‐770. 10.1016/j.clinthera.2020.03.008 32276734

[89] Konstantinou G , Konstantinou G . Psychological stress and chronic urticaria: a neuro‐immuno‐cutaneous crosstalk. A systematic review of the existing evidence. Clin Ther. 2020;42(5):771‐782. 10.1016/j.clinthera.2020.03.010 32360096

[90] Hahad O , Lelieveld J , Birklein F , Lieb K , Daiber A , Münzel T . Ambient air pollution increases the risk of cerebrovascular and neuropsychiatric disorders through induction of inflammation and oxidative stress. Int J Mol Sci. 2020;21(12):4306. 10.3390/ijms21124306 32560306 PMC7352229

[91] Taylor A , Davies N , Ware J , VanderWeele T , Smith G , Munafò M . Mendelian randomization in health research: using appropriate genetic variants and avoiding biased estimates. Econ Hum Biol. 2014;13(100):99‐106. 10.1016/j.ehb.2013.12.002 24388127 PMC3989031

[92] Burgess S , Davey SG , Davies N , et al. Guidelines for performing Mendelian randomization investigations: update for summer 2023. Wellcome Open Res. 2019;4:186. doi:10.12688/wellcomeopenres.15555.3 32760811 PMC7384151

